# An Evolutionary Approach for the Enhancement of Dermatological Images and Their Classification Using Deep Learning Models

**DOI:** 10.1155/2021/8113403

**Published:** 2021-07-15

**Authors:** Chaahat, Naveen Kumar Gondhi, Parveen Kumar Lehana

**Affiliations:** ^1^Department of Computer Science and Engineering, Shri Mata Vaishno Devi University, Katra 182301, India; ^2^MIET, Jammu 181122, India; ^3^Department of Electronics, University of Jammu, Jammu 180006, India

## Abstract

Dermatological problems are the most widely spread skin diseases amongst human beings. They can be infectious, chronic, and sometimes may also lead to serious health problems such as skin cancer. Generally, rural area clinics lack trained dermatologists and mostly rely on the analysis of remotely accessible experts through mobile-based networks for sharing the images and other related information. Under such circumstances, poor image quality introduced due to the capturing device results in misleading diagnosis. Here, a genetic-algorithm- (GA-) based approach used as an image enhancement technique has been explored to improve the low quality of the dermatological images received from the rural clinic. The diagnosis is performed on the enhanced images using convolutional neural network (CNN) classifier for the identification of the diseases. The scope of this paper is limited to only motion blurred images, which is the most prevalent problem in capturing of the images, specifically when any of the two (device or the object) may move unpredictably. Seven types of skin diseases, namely, melanoma, melanocytic nevus, basal cell carcinoma, actinic keratosis, benign keratosis, vascular lesion, and squamous cell carcinoma, have been investigated using ResNet-152 giving an overall accuracy of 87.40% for the blurred images. Use of GA-enhanced images increased the accuracy to 95.85%. The results were further analyzed using a confusion matrix and *t*-test-based statistical investigations. The advantage of the proposed technique is that it reduces the analysis time and errors due to manual diagnosis. Furthermore, speedy and reliable diagnosis at the earliest stage reduces the risk of developing more severe skin problems.

## 1. Introduction

Skin is the largest organ of the human body protecting us against injuries, infections, and environmental hazards. In clinical evaluation, it helps in the assessment of a patient's prime health status. Functioning of the liver, heart, and immune system may be empirically estimated from the analysis of the patient skin. Skin diseases are the most prevalent among other health issues. Skin diseases are generally categorized into degenerative, infectious, inflammatory, viral, and malignant [1]. Malignant skin diseases such as psoriasis, eczema, and melanoma may lead to fatal consequences if not timely diagnosed. Furthermore, the increase in the cases of skin cancers has been reported worldwide, especially in the United States. About 9,500 people per day in the U.S. are diagnosed with skin cancer [2]. Melanoma is the most common form of skin cancers. It is a malignant tumor of melanocytes produced due to mutations occurring within the skin [3]. The main cause of the occurrence of melanoma is the continuous high-intensity exposure to Ultraviolet (UV) radiations. Sometimes, sunburns developed during childhood may increase the chances of occurrence of the melanoma [4]. According to the surveys, about 87110, 91270, and 192310 patients were reported to be suffering from melanoma in America during 2017, 2018, and 2019, respectively [5–7]. The American Cancer Society has predicted that melanoma cases would rise to 100350 by the end of 2020 and will result in death of about 6,850 patients in America alone [3]. Similar cases have also been reported in Australia and Europe [8, 9].

Accurate timely diagnosis of skin diseases can rarely be achieved in rural areas due to poor availability of resources including well-trained domain experts. In these areas, either patients or their clinical samples are sent for diagnosis to the experts in urban areas, which can be quite time consuming, and sometimes, the delay may lead to serious problems. One of the solutions for reducing the delay and enhancing the accuracy of the diagnosis may be using mobile-based applications for capturing and sending the skin images to experts in well-equipped catheterization labs in urban cities.

The problem associated with images of skin captured using a mobile is that it introduces some blurredness, reducing the capability of visual analysis. This can be tackled by automatically enhancing and classifying the captured images using nature-inspired evolutionary algorithms, such as Genetic Algorithm (GA) and Convolution Neural Networks (CNNs), respectively. In this paper, GA has been employed as a preprocessing technique for enhancing the low-quality blurred dermatological images, followed by CNN-based diagnosis or classification.  Section 2 gives the related work.  Section 3 discusses the proposed methodology for GA-based enhancement, CNN classifier, and the investigations carried out.  Section 4 presents the results of the investigations, and Section 5 is devoted to conclusions along with the future work.

## 2. Related Work

This section includes relevant works in convolutional-neural-network-based classification of skin lesions, image blurring mechanisms, and genetic algorithm. CNNs are a subset of neural networks using mathematical convolutional operation instead of deriving parameters by simple multiplication as used in common neural network architectures. CNNs use a multiple-layer approach for machine learning. The concept of CNN was introduced by Krizhevsky et al. [9] during investigations with the ILSVRC dataset for image classification applications. In general, a CNN is a hierarchical neural network consisting of the convolutional layers, pooling layers, and fully connected layers [10, 11], as shown in Figure 1. CNNs have found their applications in various fields, especially in dermatology [12–18].

Pixel-based seed segmented image fusion for automatic detection and classification of melanoma was investigated by Rehman et al. [19]. In the technique, contrast stretching, fusion-based lesion segmentation, and multilevel feature extraction followed by classification using support vector machine were employed for melanoma classification with accuracy above 90%. Similar work has been carried out by Nasir et al. [20]. In [21], for localization and recognition of skin cancer lesions, an automated Newton–Raphson-based deep feature selection method with a deep learning model has been reported. Classification accuracy using ISBI 2016 and ISBI 2017 datasets was reported as 94.5% and 93.4%, respectively.

Recently, Artificial Intelligence (AI), Computer Vision (CV), Deep Learning (DL), Machine Learning (ML), and particularly, convolution neural networks have been employed successfully for identification and classification of diseases from images obtained from different sources such as MRI, CT scan, ultrasound, and digital cameras [22–24]. The main limitation of these techniques is the computational complexity and requirement of a huge dataset for training. Mostly available datasets are limited in size, and hence, transfer-based learning is generally preferred. Another problem with the medical images may be the distortions introduced because of the variations in lighting conditions, resolution of the acquiring devices, rotation angles, scaling, and other manufacturer-dependent limitations of the capturing devices. Some of these limitations may be compensated by the use of preprocessing of the images obtained by the various sources [25].

There are several types of blurring mechanisms present in the optical system and the environment [26]. In blurred images, the mechanism involves more than one blurring basic submechanism. In most of the cases, the blurring can be attributed to the undesired movement of the optical system of the capturing devices. In [26], the authors have conducted experiments with Gaussian blur filters and concluded this method is better over other techniques such as bilateral-filter-based methods. Investigations involving depth-based blurring of images are reported in [27], and blurring based on environmental parameters has been reported in [28].

Classification of skin lesions using the CNN has been successfully carried out by Yu et al. [29] taking dermoscopy images of acral melanoma and benign nevi. A total of 724 images (350 acral melanoma) and (374 benign nevi) were used in the investigations, giving an accuracy of more than 80% for the classification of the skin diseases. Zhang et al. [30] reported more than 87% accuracy for classification of seborrheic keratosis, psoriasis, melanocytic nevus, and basal cell carcinoma using a dataset consisting of 1067 images. Delibasis et al. [31] investigated a prefiltering-based skin lesion characterization using deep transfer learning and reported the enhancement in classification accuracy of melanoma from 70% to 77%.

Preprocessing followed by neural-network-based classifier showed an accuracy of 95%. Sultana et al., using a regularized discriminant CNN-based framework for melanoma, reported an accuracy of 73.8%, 98.5%, 68.8%, and 78.83% for four standard medical datasets (ISBI 2016, ISBI 2017, PH2, and MED-NODE) [32]. Alam et al. [33] reported an identification accuracy of 80% for mild eczema and 93% for severe eczema on the basis of texture using a severity index tool. Accuracy more than 97% has been also reported by Albahar [34] for the classification of the skin lesions using binary regularized classifier. AlexNet, VGG, GoogLeNet, and ResNet models have been successfully investigated for the classification of skin lesions.

The accuracy of the classification of skin diseases is highly dependent upon the quality of the input images. Several techniques such as unsharp masking, pyramid recombination, homomorphic filtering, dynamic histogram equalization, multiscale adaptive histogram equalization, wavelet, orthogonal, and homological transform techniques have been attempted for the enhancement of input images [35–37]. The main limitations of these techniques are digitization effect, noise amplification, underenhancement, and overenhancement. To compensate these limitations, optimization techniques are used. They provide the optimum solution out of all the possible outcomes. Genetic algorithm (GA) is one of the best optimization approaches giving promising results under multiple constraints. Introduced by John Holland, GA mimics the process of biological evolution of the nature discovered by Charles Darwin [38]. Since the last decade, GA has been effectively used in image enhancement, feature extraction, segmentation, classification, and image reconstruction [39].

The basic operations of GA are selection, crossover, and mutation. In genetic algorithm, population is a set of chromosomes, each indicating a possible solution to the given problem. Each chromosome is associated with a fitness function capable of ranking a particular solution against all the available possibilities. The fitness score helps in the selection of the individuals for reproduction. Selection is analogous to the concept of the survival of the fittest. Various techniques to implement selection are tournament, roulette wheel, rank, and steady-state selections [38]. After applying the selection operation, crossover randomly chooses two chromosomes with predefined priorities. Mutation introduces some random changes in the offspring chromosomes to maintain the diversity in the solution space. The number of iterations required for the final solution depends upon the convergence of the intermediate results. GA is useful for problem solving associated with huge and complex datasets. The main advantage of GA is that it requires less prior information about the problems to be solved [39].

Munteanu and Rosa [40] observed that better results could be obtained using GA in comparison to other methods such as histogram equalization and linear stretching. Superiority of GA has also been reported in [41] for the enhancement of natural images captured in poor lighting conditions using ten randomly initialized DNAs over 1000 successive iterations, and a quality index of 0.2 was reported. GA has also been used for developing an input-output relation between their gray levels for enhancing the contrast of the given images [42].

## 3. Proposed Methodology

Overall workflow of the proposed system for analysis and diagnosis of dermatological diseases is shown in Figure 2. A health worker at a rural clinic center captures the patient's skin lesion using some mobile application. The images are transferred over the mobile network to the well-equipped catheterization lab which may be situated in some urban area. Prior to diagnosis using the CNN, the received images are enhanced using GA-based algorithm as the quality of the images may generally be low because of unpredictable errors introduced at the rural clinic such as random movement of the device or the patient. The classified images are sent to the domain experts for analysis and report preparation. Furthermore, the database is also updated as per the feedback received from the experts, and the final analysis report is sent to the rural clinic center. The CNN is retrained regularly in accordance with the updated information from the domain experts. The scope of this paper is limited to investigations related to GA enhancement capability and CNN classification efficiency for accurate diagnosis of the skin disease. For training, a publically available dataset (International Skin Imaging Collaboration 2019 challenge) [43–45] has been used. The dermatofibroma class from this dataset has not been taken for investigations as it did not give satisfactory results during preanalysis. To simulate the effect of unpredictable movement caused by motion blurring using (1), 589 test images were randomly taken from the dataset such that each of the seven classes was adequately considered, as represented in Table 1.

(1) $$\begin{array}{c} h=f\left(p_{m},l,\theta \right), \end{array}$$

where *h* represents a set of filter coefficients to be used for blurring by convolving it with the input image. The type of relative motion of the capturing device is specified by *p*_*m*_, *l* specifies the length of the motion, and *θ* defines the angle of motion in degrees in a counterclockwise direction [46]. The value of length has been varied in the range 9 to 100 and that of theta from 0 to 5 degrees.

For the GA-based investigations, these blurred test images were used as input. The chromosome structure used in GA enhancement with various parameters is shown in Figure 3, where type specifies the filter, hsize refers to the filter size, radius represents the influential filter area, sigma represents the standard deviation, and alpha represents the Laplacian shape. The remaining parameters length and theta have already been explained. Equivalent vector representation of these parameters is also shown in Figure 4.

An initial population of ten chromosomes was randomly generated. Fitness value (or image quality) was calculated for each chromosome. Naturalness image quality evaluator (NIQE) has been used for intermediate quality assessment. It evaluates the quality of the image based on the natural scene statistics model [47]. Smaller score indicates better perceptual quality. These fitness values obtained in each iteration for every chromosome were sorted in descending order. The length parameter of the chromosome was chosen as the crossover point for generating new offsprings. The mating was carried out using random combinations of the chromosomes from the whole population. For mutation, one random candidate from the best 80% population was randomly selected. The algorithm was run for about 1000 generations for each blurred image.

Overall, for investigating the classification accuracy using the CNN (ResNet-152) [40], the blurred images given to the GA as input and the corresponding enhanced one by the GA were separately applied to the CNN for classification. Quantification of the accuracy of classification of the CNN was estimated using a confusion matrix and *t*-test-based statistical analysis.

## 4. Experimental Results and Discussion

The quality of the original, motion-blurred dermatological disease images and that of their intermediate images obtained during GA-based processing has been discussed in this section. The investigations showed that about 1000 generations are adequate for achieving satisfactory quality of the blurred images. GA-enhanced and their corresponding blurred image datasets were further sent to RESNET-152 for their classification in their respective classes. Figures 5to 11 show the results of GA-based enhancement for different dermatological diseases.

The results for melanoma are presented in Figure 5. The quality of the original image (Figure 5(a)) was obtained as 3.43, and that of the motion-blurred image (Figure 5(b)) using parameters (19, 3) was 5.06. After 55 iterations using the GA approach, the image showed some improvement in fitness score as 4.82. The adapted chromosome after these generations was [7.00, 7.00, 5.00, 0.20, 0.50, 19.54, 2.89]. It may be seen from the image (Figure 5(c)) that there is some enhancement of the quality. After 75 iterations (Figure 5(d)), the chromosome adapted to [8.00, 6.00, 10.00, 0.60, 0.50, 19.02, 2.98] leading to a fitness score value of 3.50.

The investigations showed that, after 100 iterations (Figure 5(e)), the quality stabilizes to 3.42 and the chromosome to [3.00, 6.00, 10.00, 0.70, 0.20, 19.18, 3.00]. It may be noted that the final fitness score approaches to the quality of the original image, but the change from iteration to iteration is not appreciably visible in the processed images.

Analysis of melanocytic nevus is presented in Figure 6. The quality of the original image (Figure 6(a)) was 2.78, whereas that of the motion-blurred image (Figure 6(b)) using parameters (20, 1) was 5.30. The GA-based approach showed negligible enhancement even after 25 iterations (Figure 6(c)), and the quality score achieved was just 5.24. The chromosome after these iterations was [7.00, 3.00, 4.00, 0.70, 0.10, 29.00, 0.00]. After 55 iterations (Figure 6(d)), the chromosome adapted to [4.00, 5.00, 5.00, 0.30, 0.40, 20.65, 0.93], thus improving the image quality and generating a fitness score value of 3.23. Further analysis after 100 generations (Figure 6(e)) showed that the image quality approaches to 2.77 which is almost the same as that of the original image, and the chromosome generated for this iteration was [5.00, 6.00, 10.00, 0.10, 0.20, 20.39, 1.00].

The results for basal cell carcinoma are shown in Figure 7. The original image (Figure 7(a)) quality was 3.31, and that of the motion-blurred image (Figure 7(b)) using parameters (19, 3) was estimated as 6.03. After 25 iterations, very less improvisation is observed (Figure 7(c)) having a fitness score of 5.41. The adapted chromosome was [4.00, 5.00, 2.00, 1.00, 0.20, 17.70, 2.97]. After 38 iterations (Figure 7(d)), the chromosome modified to [5.00, 5.00, 4.00, 0.60, 0.10, 19.20, 3.05] and fitness score to 3.50. Investigations showed that, after 100 iterations (Figure 7(e)), the quality becomes stable near to 3.41 and the chromosome to [5.00 5.00, 4.00, 0.60, 0.10, 19.20, 2.97].

The results for actinic keratosis are presented in Figure 8. The quality of the original image (Figure 8(a)) was obtained as 3.49, and that of the motion-blurred image (Figure 8(b)) using parameters (16, 2) was 6.71. After 7 iterations (Figure 8(c)), the image shows improvement in fitness score giving it as 4.77 leading to a somewhat enhanced image, and the chromosome adapted to [1.00, 7.00, 1.00, 0.40. 0.50, 16.00, 1.00]. It adjusted to [1.00, 7.00, 1.00, 0.40, 0.50, 16.00, 2.02] along with a fitness score of 3.54 after 20 iterations (Figure 8(d)). After 100 iterations (Figure 8(e)), the quality approaches to 3.50 and the chromosome to [1.00, 7.00, 1.00, 0.40, 0.50, 16.00, 2.00].

The results for benign keratosis are shown in Figure 9. The original image (Figure 9(a)) quality was 3.58, and that of the motion-blurred image (Figure 9(b)) using parameters (16, 2) was 5.24. After 20 iterations, the image (Figure 9(c)) shows some improvement in the image giving a fitness score of 4.66 and the chromosome was [7.00, 6.00, 9.00, 0.50, 0.10, 16.43, 1.32]. The chromosome adapted to [6.00, 5.00, 1.00, 0.90, 0.50, 16.77, 2.06] after 50 iterations (Figure 9(d)), reaching to an image quality of 3.78. After 100 iterations (Figure 9(e)), the quality stabilizes to 3.59 and the chromosome to [6.00, 7.00, 1.00, 1.00, 0.30, 16.98, 2.00].

The results for vascular lesion are presented in Figure 10. The quality of the original image (Figure 10(a)) was 2.99, and that of the motion-blurred image (Figure 10(b)) using parameters (15, 2) was 5.60. After 8 iterations, the fitness score obtained was 8.16 and the adapted chromosome was [6.00, 3.00, 1.00, 0.50, 0.30, 15.70, 0.00]. It may be noted that the image shows almost negligible improvement (Figure 10(c)). But, after 65 iterations (Figure 10(d)), the chromosome modified to [6.00, 3.00, 1.00, 0.50, 0.30, 15.70, 2.10] giving a score of 4.10. Further investigations showed that, after 100 iterations (Figure 10(e)), the quality stabilizes to 3.43 and the chromosome to [1.00, 4.00, 7.00, 0.40, 0.50, 15.14, 1.93]. The important point to note in this case is that the quality does not stabilize within 100 iterations but takes several more iterations to become satisfactory.

The results for squamous cell carcinoma are shown in Figure 11. The quality of the original image (Figure 11(a)) was 3.86, and that of the motion-blurred image (Figure 11(b)) using parameters (20, 1) was 5.63. After 30 iterations, the image (Figure 11(c)) shows no significant improvement, but after 50 iterations (Figure 11(d)), the fitness score settles around 3.50 with the chromosome vector near [1.00, 5.00, 1.00, 0.80, 0.20, 20.83, 0.91]. After 100 iterations (Figure 11(e)), the quality further improves, giving the score of 3.42 along with the chromosome vector of [3.00, 6.00, 10.00, 0.70, 0.20, 19.18, 3.00]. The analysis shows that the proposed method efficiently improves the quality of the motion-blurred images.

The analysis based on confusion matrices (Figures 12 and 13) also supports this conclusion as the diagonal elements in the GA-enhanced matrix (Figure 12) are greater than the corresponding elements in the motion-blurred matrix (Figure 13), indicating superiority of the proposed technique.

The results of CNN-based classification are presented in Tables 2 and 3. The results have also been graphically represented in Figures 14 and 15.  Table 2 lists the individual class accuracy. The classification accuracy for GA-processed images varies from 84.62% (vascular lesion) to 99.50% (melanocytic nevus). In case of blurred images, the maximum accuracy (96.88%) was obtained for basal cell carcinoma and minimum (60.87%) for squamous cell carcinoma. Relatively more standard deviation, i.e., 11.86, was obtained for blurred images in comparison to 5.97 for GA-enhanced images around their mean values of 82.35 and 93.65, respectively. The reasons of the variations in the classification accuracy may be due to less number of available images for a particular disease or similarity among the visual patterns of the diseases.

Table 3 presents the overall classification accuracy of the CNN, and the same is graphically represented in Figure 15. The overall accuracy is defined as the ratio of correctly classified images to the total number of input images [39].

For estimating statistical significance, two-tailed paired *t*-test analysis was also carried out, as in Table 3, with the following hypothesis.

Null hypothesis (i.e., the mean of GA-enhanced and blurred images is the same):

(2) $$\begin{array}{c} H_{0}:\mu_{1}-\mu_{2}=0. \end{array}$$

Alternate hypothesis (i.e., significant enhancement has been introduced by the proposed technique):

(3) $$\begin{array}{c} H_{a}:\mu_{1}-\mu_{2}>0. \end{array}$$

The sample mean *d* = 11.30, standard deviation *s* = 8.13, sample size *n* = 7, degree of freedom d*f* = 6, and the *t* value 3.68. As the *p* value (0.005) comes out to be less than the significance level (0.05), the null hypothesis gets rejected leading to the conclusion that the proposed technique is significantly effective for enhancing the input dermatological images.

## 5. Conclusions and Future Work

An automated image enhancement followed by a CNN-based skin lesion diagnosis has been implemented and investigated for applications in resource-poor environments such as rural areas. Investigations showed the ResNet-152-based system is able to enhance the classification accuracy from 87.40% to 95.85% when GA-enhanced images are used for diagnosis. The GA-based enhancement was able to improve the blurred images to a satisfactory level. Use of additional datasets and implementation of the complete system for rural areas is on our future plan.

This work is licensed under a Creative Commons Attribution 4.0 International License, which permits unrestricted use, distribution, and reproduction in any medium, provided the original work is properly cited.

## Figures and Tables

**Figure 1:** Architecture of the convolution neural network.

**Figure 2:** Proposed methodology architecture.

**Figure 3:** Chromosome structure for GA-based image enhancement.

**Figure 4:** Vector representation of chromosome parameters.

**Figure 5:** Genetic-algorithm-based processing of dermatological images corresponding to the melanoma disease category taken from the head region of a 35-year-old male subject: (a) the original image, (b) modified image using motion blurring with parameters (length = 19, theta = 3), (c) GA-processed image after 55 generations, (d) GA-processed image after 75 generations, and (e) GA processed image after 100 generations.

**Figure 6:** Genetic-algorithm-based processing of dermatological images corresponding to the melanocytic nevus disease category taken from the lower extremity of a 10-year-old female subject: (a) the original image, (b) modified image using motion blurring with parameters (length = 20, theta = 1), (c) GA-processed image after 25 generations, (d) GA-processed image after 55 generations, and (e) GA-processed image after 100 generations.

**Figure 7:** Genetic-algorithm-based processing of dermatological images corresponding to the basal cell carcinoma disease category taken from the neck area of a 45-year-old female subject: (a) the original image, (b) modified image using motion blurring with parameters (length = 19, theta = 3), (c) GA-processed image after 25 generations, (d) GA-processed image after 38 generations, and (e) GA-processed image after 100 generations.

**Figure 8:** Genetic-algorithm-based processing of dermatological images corresponding to the actinic keratosis disease category taken from the neck region of an 80-year-old male subject: (a) the original image, (b) modified image using motion blurring with parameters (length = 16, theta = 2), (c) GA-processed image after 7 generations, (d) GA-processed image after 20 generations, and (e) GA-processed image after 100 generations.

**Figure 9:** Genetic-algorithm-based processing of dermatological images corresponding to the benign keratosis disease category taken from the anterior torso of a 55-year-old male subject: (a) the original image, (b) modified image using motion blurring with parameters (length = 16, theta = 2), (c) GA-processed image after 20 generations, (d) GA-processed image after 50 generations, and (e) GA-processed image after 100 generations.

**Figure 10:** Genetic-algorithm-based processing of dermatological images corresponding to the vascular lesion disease category taken from the head region of a 75-year-old male subject: (a) the original image, (b) modified image using motion blurring with parameters (length = 15, theta = 2), (c) GA-processed image after 8 generations, (d) GA-processed image after 65 generations, and (e) GA-processed image after 100 generations.

**Figure 11:** Genetic-algorithm-based processing of dermatological images corresponding to the squamous cell carcinoma image category taken from the head region of an 80-year-old female subject: (a) the original image, (b) modified image using motion blurring with parameters (length = 20, theta = 1), (c) GA-processed image after 30 generations, (d) GA-processed image after 50 generations, and (e) GA-processed image after 100 generations.

**Figure 12:** Confusion matrix for GA-enhanced images. The true class type is shown along the *Y*-axis and the predicted one along the *X*-axis. The number in a cell (*i*, *j*) represents the prediction of the *i*th disease as the *j*th disease, taking the topmost left cell as (1, 1). For example, 4 in (4, 5) represents that the disease melanoma is predicted incorrectly as melanocytic nevus in 4 test cases out of 130 total images in the melanoma class.

**Figure 13:** Confusion matrix for motion-blurred images. The true class type is shown along the *Y*-axis and the predicted one along the *X*-axis. The number in a cell (*i*, *j*) represents the prediction of the *i*th disease as the *j*th disease, taking the topmost left cell as (1, 1). For example, 119 in (4, 4) represents that the disease melanoma is predicted accurately as melanoma in 119 test cases out of 130 total cases in melanoma.

**Figure 14:** Classification accuracy of the individual classes (%).

**Figure 15:** Overall classification accuracy of the GA-enhanced and motion-blurred images (%).

**Table 1:** Detail of the images used for testing of the proposed technique.

Classes	No. of test images
Actinic keratosis	40
Basal cell carcinoma	128
Beningn keratosis	54
Melanoma	130
Melanocytic nevus	201
Squamous cell carcinoma	23
Vascular lesion	13
Total	**589**

**Table 2:** Classification accuracy of the individual classes (%).

Classes	Images	
	GA enhanced	Blurred
Melanoma	94.62	91.54
Melanocytic nevus	99.50	87.56
Basal cell carcinoma	99.22	96.88
Actinic keratosis	92.50	77.50
Benign keratosis	98.15	85.19
Vascular lesion	84.62	76.92
Squamous cell carcinoma	86.96	60.87

**Table 3:** Overall classification accuracy of the GA-enhanced and motion-blurred images (%).

Images	Overall accuracy
GA enhanced	95.85
Motion blurred	87.40

## Data Availability

Datasets analyzed in this study are publicly available. These data can be found at https://challenge2019.isic-archive.com/data.html.
